RETRACTED

# Correlation between 24-Hour Ambulatory Blood Pressure Variability and White Matter Lesions in Patients with Cerebral Small Vascular Disease: A Cross-Sectional Study

**DOI:** 10.1155/2022/6364769

**Published:** 2022-08-08

**Authors:** Ping Liu, Changhao Yin, Meilingzi Liu, Lu Chang, Tianjiao Wu, Zihao Li, Ruidi Luo, Xiao Du, Weina Zhao

**Affiliations:** ^1^Department of Neurology, Hongqi Hospital Affiliated to Mudanjiang Medical University, Mudanjiang, China; ^2^Heilongjiang Key Laboratory of Ischemic Stroke Prevention and Treatment, Mudanjiang, China

## Abstract

**Objective:**

The goals of this study are to assess the correlation between 24-hour ambulatory blood pressure (BP) variability and white matter lesions (WML) in patients with cerebral small vascular disease (CSVD) and to provide guidance for the prevention of WML.

**Methods:**

A total of 136 patients diagnosed with CSVD and essential hypertension were recruited and divided into two groups. The Fazekas scale was used to quantify the severity of WML. The basic information, BP levels, BP variability, and circadian rhythm changes across these groups were recorded and compared.

**Results:**

The control group consisted of 40 subjects without WML (Fazekas score = 0), and the WML group was composed of 96 patients with WML (Fazekas score ≥ 1). Patients in the WML group were then divided into three subgroups: mild WML (*n* = 43, Fazekas score = 1), moderate WML (*n* = 24, Fazekas score = 2), and severe WML (*n* = 29, Fazekas score = 3–4). Age, history of diabetes, and serum uric acid levels were significantly increased between the WML and control groups (*P* < 0.05). The levels of 24-hour mean diastolic BP (*F* = 3.158, *P* = 0.026) and daytime mean systolic BP (*F* = 3.526, *P* = 0.017) were significantly increased between the control and WML groups. There was no significant difference in the rhythmic classification of BP among all groups (*P* > 0.05). An ordered multinomial logistic regression analysis revealed that age, triglyceride levels, and nondipper BP were independent risk factors in WML.

**Conclusion:**

Age, history of diabetes, serum uric acid levels, 24-hour mean systolic level, and daily mean systolic BP level were significantly increased between the WML and control groups. Age, triglyceride levels, and nondipper BP were independent risk factors in WML in patients with CSVD, while the 24-hour dynamic blood pressure standard deviation and 24-hour dynamic blood pressure coefficient of variation were not associated with the occurrence of WML.

## 1. Introduction

Cerebral small vessel disease (CSVD) is a common and potentially destructive subclinical disease characterized by insidious onset, slow progress, and sometimes acute attacks. The manifestations of CSVD detected by magnetic resonance imaging (MRI) include lacunar infarction, lacunes, white matter lesions (WMLs), enlarged perivascular space, and cerebral microbleeds [1]. WML refers to nonspecific, spot-like, or patch-like changes in the lateral ventricles or subcortical structures caused by multiple reasons and mainly manifest as low-signal intensity or isointensity on T1-weighted magnetic resonance images and high-signal intensity on T2-weighted magnetic resonance images and fluid-attenuated inversion recovery images [2]. WMLs are considered to be the most common lesions in elderly CSVD patients. Approximately 50%–98% of the elderly, 67%–98% of stroke patients, and 28.9%–100% of cases with Alzheimer's disease exhibit WML at various degrees [3]. The high incidence of WML suggests an urgent need to identify underlying risk factors.

RETRACTED

WMLs are associated with many factors, including age, diabetes, hypertension, smoking, drinking, hyperhomocysteinemia, decreased left ventricular diastolic function, carotid artery intima-media thickness, vitamin D deficiency, renal insufficiency, and metabolic disorders [4–8]. As an important risk factor in WML, hypertension may lead to arteriolosclerosis in the areas of WML, vascular autonomic dysfunction, and brain lesions affected by low perfusion [9]. Blood pressure (BP) variability has been reported to significantly damage the target organs of hypertensive patients, resulting in poor long-term overall prognosis [10]. Ambulatory blood pressure monitoring (ABPM) is an important diagnostic and monitoring tool for the management of hypertension as it can accurately detect the BP levels and BP variability. If the BP remains high for a long time, large fluctuations in systolic BP may occur, suggesting that systolic BP may be an independent risk factor in WML.

In view of the characteristics of CSVD, high incidence and low diagnosis rate, and the high proportion of WML in CSVD, this study focused on WML in CSVD. Hypertension is the most significant risk factor for CSVD, and ambulatory blood pressure variability is more responsive to blood pressure changes and its impact on disease than office blood pressure. Therefore, we aimed to investigate the correlation between ambulatory BP variability and WML in patients with CSVD and essential hypertension. These results may provide guidance for clinical BP control and the prevention of WML in patients with CSVD and primary hypertension.

## 2. Materials and Methods

### 2.1. Subjects

A total of 136 consecutive patients diagnosed with essential hypertension and hospitalized for CSVD in the Department of Neurology of our hospital between October 2019 and December 2020 were recruited to participate in this study. All subjects were evaluated for study eligibility prior to enrollment.

RETRACTED

The inclusion criteria were as follows: (1) aged between 35 and 80 years; (2) diagnosed with essential hypertension according to the 2018 Chinese Guidelines for Prevention and Treatment of Hypertension-A report of the Revision Committee of Chinese Guidelines for Prevention and Treatment of Hypertension [11]; (3) met the diagnostic criteria of hypertension under 24-hour ABPM (average systolic BP/diastolic BP ≥ 130/80 mmHg for 24 hours; average systolic BP/diastolic BP ≥ 135/85 mmHg during the day; average systolic BP/diastolic BP ≥ 120/70 mmHg at night); (4) diagnosed with CSVD according to the Consensus on the Diagnosis and Treatment of Cerebral Small Vascular Disease^2^; (5) with full awareness and willingness to participate. Patients were excluded if they were (1) previously diagnosed with other diseases that may cause hypertension, such as kidney disease, cardiovascular disease, endocrine diseases (e.g., pheochromocytoma, Cushing's syndrome, primary aldosteronism); (2) with clear causes of WML, such as carbon monoxide poisoning, immune-mediated white matter demyelination, metabolic diseases, or genetic diseases; (3) with other disorders that might affect BP levels, such as mental problems. All patients provided written informed consent before the study and continued to take their routine medications throughout their participation.

### 2.2. Patient and Public Involvement

Participants were all hospitalized patients after outpatient visits. Patients who met the inclusion criteria would write informed consent from each subject before enrollment. Patients and the public will not be involved in the development of the research question or the design of the study. Patients will not be involved in the recruitment of participants or the conduct of the study. The general results would be disseminated to participants through public education activities.

### 2.3. Collection of Basic Information

The basic information of all recruited patients was collected from medical records, including gender, age, history of smoking, history of drinking, history of diabetes, fasting blood glucose (FBG) levels, blood uric acid (UA) levels, total cholesterol (CHOL) levels, triglyceride (TG) levels, high-density lipoprotein (HDLC) levels, low-density lipoprotein (LDLC) levels, homocysteine (HCY) levels, mean platelet volume (MPV), and platelet count (PLT).

### 2.4. ABPM

All patients underwent 24-hour ABPM after the MRI examination. The ABPM cuff was placed on the nondominant arm of the patient, with the lower edge of the cuff 2 cm above the elbow. Patients were allowed to take routine medications and perform normal daily activities, but were instructed to avoid excessive or strenuous activities. BP was measured every 30 minutes during the day (from 6 a.m. to 6 p.m.) and every one hour during the night (from 6 p.m. to 6 a.m.). The ABPM results with ≥80% valid data were considered eligible for analysis. The following dynamic BP parameters were recorded: 24-hour mean systolic blood pressure (24hSBP), 24-hour mean diastolic blood pressure (24hDBP), daytime mean systolic blood pressure (dSBP), daytime mean diastolic blood pressure (dDBP), nighttime mean systolic blood pressure (nSBP), nighttime mean diastolic blood pressure (nDBP), nighttime diastolic blood pressure coefficient of variation (nDBPCV), 24-hour dynamic blood pressure standard deviation (SD), and 24-hour dynamic blood pressure coefficient of variation (CV). According to the changes in BP levels during the circadian rhythm, there were four ambulatory BP patterns: (1) dipper BP, with a 10%–20% decrease in nSBP; (2) superdipper BP, with a >20% decrease in nSBP; (3) nondipper BP, with a <10% decrease in nSBP; (4) antidipper BP: with an increase in nSBP [12, 13].

RETRACTED

### 2.5. WML Detection

A craniocerebral MRI examination, including T1-weighted imaging, T2-weighted imaging, and fluid-attenuated inversion recovery sequence, was performed during hospitalization using a 3.0 T superconducting magnetic resonance scanner. Patients were required to remain awake, quiet, and motionless during the scanning. The severity of WML was quantified using the Fazekas scale: 0, absence of lesions; 1, spot-like, inconspicuous changes surrounding the lateral ventricles; 2, visible changes surrounding the lateral ventricles; 3, irregular, continuous changes surrounding the bilateral ventricles and/or in the center of the semi-oval; 4: continuous changes surrounding the lateral ventricles and/or in the center of the semioval. Patients with a Fazekas score of 0 were categorized into the control group (*n* = 40), while those with a score of ≥1 were assigned to the WML group (*n* = 96). Patients with WMLs were further divided into three subgroups according to the severity of the WMLs: mild WML (*n* = 43, Fazekas score = 1), moderate WML (*n* = 24, Fazekas score = 2), and severe WML (*n* = 29, Fazekas score = 3–4) [14, 15].

### 2.6. Statistical Analysis

The SPSS 20.0 software was used for statistical analysis. A Levene's test was used to assess the homogeneity of the variances of different variables. Gender, history of smoking, history of drinking, history of diabetes, and ambulatory BP patterns were expressed as a number (frequency) and compared using a chi-square test. Normally distributed data, including the levels of UA, CHOL, TG, HDL, LDL, and MPV, PLT, the ratio of PLT/MPV, and ABPM parameters were presented as mean ± standard deviation (SD) and compared using the one-way ANOVA. Pairwise LSD *t*-tests were used to correct for multiple comparisons. Nonnormally distributed variables, such as the level of fasting blood glucose and HCY, were represented as the median and quartile [M(IQR)] and were compared using a Kruskal-Wallis *H* test. The risk factors were identified by single-factor logistic regression analysis, followed by ordered multinomial logistic regression analysis. A value of *P* < 0.05 was considered statistically significant.

RETRACTED

## 3. Results

### 3.1. Age, History of Diabetes, and UA Were Significantly Increased in WML

Among the 136 recruited patients, 72 (52.94%) were males. The average age of all participants was 61.58 ± 12.93 years. There were 40 cases in the control group (23 males), 43 cases in the mild WML group (24 males), 24 cases in the moderate WML group (11 males), and 29 cases in the severe WML group (14 males). There was no significant difference in gender between the control and WML groups (*P* > 0.05). Age, history of diabetes, and serum UA levels were significantly increased between the WML and control groups (*P* < 0.05). The average age of the control group was significantly lower than that of the moderate and severe WML groups (both, *P* < 0.05). The average age of the mild WML group was significantly lower than that of patients with moderate lesions (*P* = 0.023) or severe lesions (*P* = 0.012). The UA levels were significantly different between the mild and severe WML groups (*P* = 0.042) and between the moderate and severe WML groups (*P* = 0.04) (Table 1).

### 3.2. 24 h SBP and dSBP Were Significantly Increased in WML

The 24hSBP was significantly increased between the control and WML groups (*F* = 3.158, *P* = 0.026). The 24hSBP of the control group was significantly lower than that of the mild (*P* = 0.006) and severe (*P* = 0.015) WML groups. No difference in 24hSBP between other groups was observed. The dSBP was significantly increased among all groups (*F* = 3.526, *P* = 0.017). The dSBP of the control group was significantly lower than that of the mild (*P* = 0.003) and severe (*P* = 0.015) WML groups. In addition, the differences in other dynamic BP parameters such as nSBP (SD/CV), nDBP (SD/CV), 24hSBPSD, 24hDBPSD, 24hSBPCV, and 24hDBPCV between groups were not statistically significant (*P* > 0.05) (Table 2).

### 3.3. Comparison of Ambulatory BP Patterns

The ABPM results showed that there were 14 dipper hypertensive subjects, 7 superdipper hypertensive subjects, 71 cases with nondipper hypertension, and 44 cases with antidipper hypertension. The numbers of patients with different ambulatory BP patterns were not significantly different in the control group and WML groups (*χ*^2^ = 6.158, *P* = 0.724) (Figure 1).

RETRACTED

Age, TG, and nondipper BP were independent risk factors in WML The univariate logistic regression analysis showed that age (*P* = 0.004), history of diabetes (*P* = 0.004), TG levels (*P* = 0.021), and nDBPCV (*P* = 0.041) were potential risk factors in WML. The ordered multinomial logistic regression analysis that included potential influential factors (significantly different variables shown in Tables 1 and 2) and ambulatory BP patterns revealed that age (*P* = 0.018), TG levels (*P* = 0.049), and nondipper BP (*P* = 0.042) were independent risk factors in WML (Table 3).

## 4. Discussion

The present study showed that patients with WML exhibited a higher prevalence of diabetes, advanced age, and high levels of serum UA, 24hSBP, and dSBP compared to those without WML. Furthermore, the ordered multinomial logistic regression analysis after adjustment for confounders showed that age, TG levels, and nondipper BP were independent risk factors in WML in patients with CSVD.

Age has been identified as an independent risk factor for periventricular WML in British and American populations [16, 17]. Also, intracranial small vascular atherosclerosis progresses with age. In our study, after adjusting for confounders, age remained an independent risk factor in WML. Cerebrovascular hypoperfusion causes insufficient blood supply in WML and the formation of ischemic lesions. Subsequent blood-brain barrier disruption and IgG/albumin leakage in the cerebrospinal fluid can lead to microstructural changes in WML. The major structural components of WML, such as lecithin and protein-myelin basic protein, also degrade with age [18]. A study in Japan showed that TG levels were related to the occurrence, but not the progression, of WML [4]. Another study found that people with high TG levels were more susceptible to WML and that high TG levels were positively correlated with the severity of WML [19]. Here, we identified TG level as an independent risk factor in WML, which might be related to cerebral atherosclerosis caused by hyperlipidemia.

Blood pressure variability represents the degree of blood pressure fluctuation over a certain period of time, and 24 h ambulatory blood pressure variability is a cardiovascular and stroke risk factor independent of blood pressure level [20]. Elevated blood pressure and sharp fluctuations in blood pressure could lead to changes in the tension and stress of blood pressure on the vascular wall, resulting in vascular endothelial dysfunction and vascular structural damage. In addition, rapid changes in blood pressure would cause the blood pressure to drop too much, resulting in hypoperfusion of the cerebral blood. Endothelial dysfunction, ischemia, and hypoperfusion were all the pathogenesis of CSVD [21, 22]. Previous studies have demonstrated that the levels of 24hSBP and dSBP were negatively correlated with the occurrence of WML and that the increase in BP levels and blood flow volatility might aggravate small vascular atherosclerosis [23, 24]. Therefore, it was important to apply ABPM to hypertensive patients in clinical settings to determine the occurrence of WML [25, 26]. Dijk et al. found that both systolic and diastolic BP were related to the occurrence of WML [27]. However, a recent study reported that diastolic BP levels were correlated with WML scores, while systolic BP levels were not [28]. This inconsistency may be due to racial disparities and patient selection. In our study, the single-factor logistic regression analysis showed that nDBPCV might be related to WML, which was consistent with a previous study in China [29]. This work also showed that, after adjustment for confounders, the standard deviation and variability of ambulatory BP were no longer significantly correlated with WML, which might be attributed to the sample size, inclusion criteria, and scoring method.

RETRACTED

Fluctuations in BP during the circadian rhythm generally occurred within a normal range (i.e., 10%–20% decrease during sleep) and was called dipper BP. The circadian rhythm of BP played an important role in promoting the normal structure and function of blood vessels without affecting vascular elasticity. Arteriosclerosis is one of the main pathogenic mechanisms of CSVD, which reduces vascular elasticity, increases cerebral arterial pulsatility, and reduces BP buffering. When considering where WML were likely to occur, it was likely that cerebral artery insufficiency led to chronic ischemia and subsequent WML [30]. ABPM is superior to office BP measurement and home BP monitoring for recording BP at different states (i.e., active or quiet, day or night). Therefore, ABPM can provide more reliable data that can be used to analyze the relationship between BP changes and WML. Lee et al. found that the most important contributor to atherosclerosis was rhythmic changes in diurnal BP. Also, patients with nondipper BP showed more severe arteriosclerosis compared with those with dipper BP [31, 32]. Here, we identified nondipper BP as an independent risk factor in WML in patients with CSVD. The decrease in systolic BP at night is a type of protection for the cardiovascular and cerebrovascular systems. In patients with nondipper BP, the BP remains high for a long time and leads to a decrease in blood vessel elasticity and an increase in pulsatility. These patients also exhibit a greater tendency for target-organ damage (e.g., heart, brain, and kidney) as well as cardiovascular and cerebrovascular disorders compared with dipper patients.

RETRACTED

In summary, age, history of diabetes, blood UA levels, 24hSBP, and dSBP were found to be significantly different between patients with and without WML. Age, TG levels, and nondipper BP were independent risk factors in WML. In BP management for patients with CSVD and essential hypertension, it is important to maintain their BP levels within a normal range and also to monitor BP variations during the circadian rhythm. These results may provide future guidance for the prevention of WML in hypertensive patients with CSVD.

## Figures and Tables

**Figure 1:** Comparison of ambulatory BP patterns in WML patients. Data are shown as number and compared using a chi-square test. A: control group; B: mild WML group; C: moderate WML group; D: severe WML group; 1: dipper; 2: superdipper; 3: nondipper; 4: antidipper.

**Table 1:** Basic characteristics of all patients and controls.

Variable	All (*N* = 136)	Control (*N* = 40)	Mild WML (*N* = 43)	Moderate WML (*N* = 24)	Severe WML (*N* = 29)	*P*
Age	61.58 ± 12.93	55.79 ± 12.92^∗^	60.00 ± 11.12^∗∗^	67.08 ± 11.60	67.41 ± 12.84	<0.001^#^
Male	72 (52.94%)	23 (16.91%)	24 (17.65%)	11 (8.09%)	14 (10.29%)	0.749^a^
History of smoking	27 (20.22%)	7 (5.51%)	9 (6.62%)	4 (2.94%)	7 (5.15%)	0.883^a^
History of drinking	27 (19.86%)	6 (4.41%)	11 (8.09%)	3 (2.21%)	7 (5.15%)	0.452^a^
History of diabetes	30 (22.07%)	3 (2.21%)	13 (9.56%)	9 (6.62%)	5 (3.68%)	0.016^a#^
FBG	5.89 (5.25–7.15)	5.86 (5.14–6.65)	5.93 (5.37–7.05)	6.51 (5.08–9.44)	5.90 (5.23–7.03)	0.972^b^
UA	370.52 ± 117.34	406.85 ± 108.66	355.23 ± 117.74	391.38 ± 145.50	325.83 ± 84.06^∗∗∗^	0.021^c#^
CHOL	4.91 ± 1.31	5.10 ± 1.07	4.94 ± 1.60	4.84 ± 1.33	4.67 ± 1.14	0.606^c^
TG	1.90 ± 1.22	2.24 ± 1.43	1.90 ± 1.05	1.71 ± 1.10	1.59 ± 1.18	0.13^c^
HDLC	1.36 ± 0.36	1.41 ± 0.39	1.32 ± 0.37	1.38 ± 0.40	1.35 ± 0.27	0.696^c^
LDLC	2.70 ± 0.89	2.78 ± 0.67	2.79 ± 1.06	2.62 ± 0.88	2.52 ± 0.92	0.547^c^
HCY	13.45 (11.33–17.88)	13.25 (11.08–15.60)	13.20 (11.30–16.70)	13.10 (10.63–18.85)	15.40 (11.9–23.15)	0.342^b^
MPV	9.78 ± 1.30	9.63 ± 1.38	9.72 ± 1.17	10.29 ± 1.55	9.63 ± 1.10	0.20^c^
PLT	231.32 ± 81.95	246.28 ± 127.90	219.02 ± 54.39	217.17 ± 44.55	240.66 ± 52.07	0.338^c^
MPV/PLT	0.047 ± 0.019	0.046 ± 0.019	0.049 ± 0.024	0.050 ± 0.016	0.042 ± 0.011	0.368^c^

Data are shown as number (frequency), mean ± SD, or *M* (IQR). FBG: fasting blood glucose; UA: blood uric acid; CHOL: total cholesterol; TG: triglyceride; HDLC: high-density lipoprotein; LDLC: low-density lipoprotein; HCY: homocysteine; MPV: mean platelet volume; PLT: platelet count; ^a^chi-square test; ^b^Kruskal-Wallis *H* test; ^c^analysis of variance followed by LSD *t*-test. ^#^*P* < 0.05, control groups vs. WML groups; ^∗^*P* < 0.05, control groups vs. moderate WML group and severe WML group; ^∗∗^*P* < 0.05, mild WML group vs. severe WML group; ^∗∗∗^*P* < 0.05, severe WML group vs. mild WML group and moderate WML group.

RETRACTED

**Table 2:** ABPM parameters of all patients and controls.

Variable	All (*N* = 136)	Control (*N* = 40)	MILD WML (*N* = 43)	Moderate WML (*N* = 24)	Severe WML (*N* = 29)	*P*
24-hour ambulatory blood pressure levels						
24hSBP	145.35 ± 14.28	139.78 ± 14.07^∗^	148.30 ± 14.02	145.96 ± 12.15	148.17 ± 15.00	0.026^#^
24hDBP	83.60 ± 12.62	81.78 ± 11.54	84.53 ± 14.58	83.17 ± 12.49	85.07 ± 11.26	0.688
dSBP	146.38 ± 14.39	140.68 ± 14.00^∗∗^	149.98 ± 14.40	146.17 ± 11.86	149.10 ± 14.99	0.017^#^
dDBP	84.34 ± 12.88	82.35 ± 11.85	85.14 ± 14.33	83.58 ± 12.45	86.52 ± 12.55	0.571
nSBP	142.05 ± 18.69	136.00 ± 17.42	144.53 ± 19.29	142.96 ± 17.15	145.97 ± 19.56	0.097
nDBP	81.66 ± 13.23	79.65 ± 11.04	83.00 ± 16.28	81.54 ± 13.75	82.55 ± 10.59	0.687
24-hour ambulatory blood pressure SD						
24hSBPSD	15.31 ± 4.63	14.94 ± 4.34	15.45 ± 5.73	14.84 ± 3.06	16.00 ± 4.336	0.760
24hDBPSD	9.95 ± 2.66	9.84 ± 2.69	9.69 ± 2.59	9.94 ± 2.12	10.48 ± 3.13	0.662
dSBPSD	14.73 ± 4.56	14.52 ± 4.47	14.68 ± 5.64	14.62 ± 3.06	15.21 ± 4.06	0.936
dDBPSD	9.54 ± 2.76	9.55 ± 2.96	9.20 ± 2.81	9.48 ± 2.45	10.08 ± 2.71	0.630
nSBPSD	12.93 ± 5.08	13.13 ± 6.02	12.96 ± 4.58	12.75 ± 4.72	12.73 ± 4.90	0.987
nDBPSD	9.08 ± 3.97	9.50 ± 4.74	8.68 ± 3.33	9.77 ± 3.94	8.52 ± 3.78	0.541
24-hour ambulatory blood pressure CV						
24hSBPCV	0.107 ± 0.034	0.108 ± 0.032	0.107 ± 0.043	0.102 ± 0.026	0.108 ± 0.030	0.915
24hDBPCV	0.121 ± 0.034	0.122 ± 0.033	0.119 ± 0.038	0.121 ± 0.027	0.122 ± 0.035	0.979
dSBPCV	0.102 ± 0.033	0.104 ± 0.033	0.100 ± 0.040	0.100 ± 0.025	0.102 ± 0.030	0.935
dDBPCV	0.115 ± 0.037	0.118 ± 0.038	0.112 ± 0.040	0.114 ± 0.031	0.118 ± 0.036	0.908
nSBPCV	0.093 ± 0.038	0.097 ± 0.044	0.093 ± 0.038	0.091 ± 0.037	0.088 ± 0.031	0.775
nDBPCV	0.113 ± 0.051	0.121 ± 0.060	0.108 ± 0.046	0.123 ± 0.050	0.102 ± 0.045	0.302

Data are shown as mean ± SD and compared by analysis of variance followed by LSD *t*-test. 24hSBP: 24-hour mean systolic blood pressure; 24hDBP: 24-hour mean diastolic blood pressure; dSBP: daytime mean systolic blood pressure; dDBP: daytime mean diastolic blood pressure; nSBP: nighttime mean systolic blood pressure; nDBP: nighttime mean diastolic blood pressure; 24hDBPSD: 24-hour dynamic blood pressure standard deviation; 24hSBPSD: 24-hour systolic blood pressure standard deviation; 24hDBPSD: 24-hour diastolic blood pressure standard deviation; dSBPSD: daytime systolic blood pressure standard deviation; dDBPSD: daytime diastolic blood pressure standard deviation; nSBPSD: nighttime systolic blood pressure standard deviation; nDBPSD: nighttime diastolic blood pressure standard deviation; 24hSBPCV: 24-hour systolic blood pressure coefficient of variation; 24hDBPCV: 24-hour diastolic blood pressure coefficient of variation; dSBPCV: daytime systolic blood pressure coefficient of variation; dDBPCV: daytime diastolic blood pressure coefficient of variation; nSBPCV: nighttime systolic blood pressure coefficient of variation; nDBPCV: nighttime diastolic blood pressure coefficient of variation. ^#^*P* < 0.05, control groups vs. WML groups; ^∗^*P* < 0.05, control groups vs. mild WML group and severe WML group; ^∗∗^*P* < 0.05, control groups vs. mild WML group and severe WML group.

RETRACTED

**Table 3:** Analysis of risk factors in WML.

Variable	Regression coefficient	Standard error	Wald *χ*^2^	*P*	95% confidential interval
Age	1.089	0.461	5.580	0.018	0.186–1.993
UA	-0.499	0.681	0.537	0.464	-1.835–0.836
TG	-0.883	0.448	3.881	0.049	-1.761–-0.005
History of diabetes	-0.452	0.494	0.838	0.360	-1.419–0.516
Dipper	-0.698	0.765	0.834	0.361	-2.197–0.801
Superdipper	-0.421	1.054	0.160	0.689	-2.486–1.644
Nondipper	0.923	0.455	4.121	0.042	0.032–1.814
24hSBP	-0.153	0.474	0.104	0.747	-1.081–0.775
dSBP	0.007	0.655	≤0.001	0.992	-1.277–1.291
nDBPCV	2.267	6.034	0.141	0.707	-9.559–14.093

UA: blood uric acid; TG: triglyceride; 24hSBP: 24-hour mean systolic blood pressure; dSBP: daytime mean systolic blood pressure; nDBPCV: nighttime diastolic blood pressure coefficient of variation.

## Data Availability

The data used to support the findings of this study are available from the corresponding author upon request.

## Additional Points

*Reporting Checklist*. The authors had completed the MOOSE reporting checklist. *Data Sharing*. No additional data available.
